The article "LncRNA MALAT1 acts as an oncogene in multiple myeloma through sponging miR-509-5p to modulate FOXP1 expression" was retracted in 2026. Reasons: plagiarized images; duplicated images; overlap with other authors' work; original data or images not available.

# LncRNA MALAT1 acts as an oncogene in multiple myeloma through sponging miR-509-5p to modulate FOXP1 expression

**DOI:** 10.18632/oncotarget.21957

**Published:** 2017-10-23

**Authors:** Yueli Gu, Xichun Xiao, Shuo Yang

**Affiliations:** ^1^ Department of Hematology, The First People's Hospital of Shangqiu, Shangqiu 476100, China

**Keywords:** multiple myeloma, ceRNA, MALAT1, miR-509-5p, forkhead box P1

## Abstract

Previous studies showed that Metastasis associated lung adenocarcinoma transcript 1(MALAT1) acted as an oncogene in Multiple Myeloma (MM). However, the underlying mechanism of MALAT1 in MM remains unclear. Quantitative real time-PCR(qRT-PCR) was used to determine MALAT1 expression in MM samples and cell lines. *in vitro* function assays were used to determine the function of MALAT1 on MM cells. Bioinformatics tools were used to predict the targets of MALAT1 and miR-509-5p, respectively. Furthermore, rescue experiments were performed to further confirm the regulation of miR-509-5p by MALAT1. In the present study, our data showed that MALAT1 expression was upregulated in MM samples and cell lines. In function assays, we confirmed that MALAT1 inhibition significantly suppressed cells proliferation, induced cells apoptosis, arrested cells in G1/S phase, and inhibited MM cells growth *in vivo*. Furthermore, MALAT1 was identified to function as a competitive endogenous RNA (ceRNA) for miR-509-5p to promote MM cell viability. Additionally, our results suggested that miR-509-5p targeted the 3’-UTR of FOXP1 to suppress MM cells progression. Meanwhile, our results showed that miR-509-5p inhibitors significantly abrogated the decreased expression of FOXP1 induced by MALAT1 suppression, indicating that MALAT1 could positively regulate FOXP1 expression by sponging miR-509-5p. Our findings suggested that MALAT1/miR-509-5p/FOXP1 axis was one of the key signalings in mediating MM cell growth, and further indicated that MALAT1 could act as a novel diagnostic marker and therapeutic target for the treatment of MM.

## INTRODUCTION

Multiple myeloma (MM) is a malignant plasma-cell (PC) disorder and clinically defined when a PC neoplasm results in clinical complications [1]. MM accounts for approximately 1% of neoplastic diseases and 13% of all hematologic cancers [2]. The disease is characterized by clonal proliferation of malignant plasma cells in the bone marrow, monoclonal para protein in blood/urine, and related organ dysfunction [3]. Despite significant progress in elucidation of the biology and treatment options over the past few decades, myeloma remains incurable, and the five-year survival rate of MM is about 40% [4]. Thus, it is urgent to investigate novel functional molecular and therapeutic targets for the treatment of MM.

Long non-coding RNAs (lncRNAs) which are defined as being longer than 200 nucleotides without or with limit protein coding ability [5]. With the help of improvements in modern biotechnology such as high-throughput sequencing and microarray analysis, growing evidence indicated that lncRNA participated in a surprisingly diverse collection of biological progress and gene regulatory events, rather than simply being leaky transcription noise as initially considered [6, 7]. Moreover, increasing studies suggested that dysregulated expressions of lncRNA occur in various diseases and might contribute to cancer biology [8]. For example, Huang et al showed that lncRNA PVT1 was upregulated in pancreatic cancer tissues and associated with patient's prognosis [9]. Li et al showed that overexpression of lncRNA HOTTIP increased chemoresistance of osteosarcoma cells by activating the Wnt/β-catenin pathway [10]. Cui et al revealed that lncRNA SNHG1 contributed to the progression of non-small cell lung cancer through inhibition of miR-101-3p and activation of Wnt/β-catenin signaling pathway [11]. However, the functional role and underlying mechanism of MALAT1 in MM remains unclear.

In this study, our data showed that upregulation of MALAT1 was a characteristic molecular change in MM, and high expression of MALAT1 was associated with clinical progression and poor overall survival of MM patients. Function assays showed that MALAT1 inhibition suppressed cell proliferation both *in vitro* and *in vivo*. Furthermore, we predicted and identified miR-509-5p as a downstream target of MALAT1. In addition, FOXP1 was demonstrated to be a direct target of miR-509-5p and acted as an oncogene in MM progression. Taken together, these data suggested that MALAT1 modulated MM cells growth via targeting miR-509-5p/FOXP1 axis.

## RESULTS

### LncRNA MALAT1 was increased in MM samples and cell lines

To determine the role of MALAT1 in MM, we determined the expression of MALAT1 in MM patients (n=37) and normal healthy controls (n=19) by qRT-PCR. The results revealed that MALAT1 expression was significantly upregulated in MM patients compared to normal healthy controls (Figure 1A; P<0.05). Besides, we evaluated the expression of MALAT1 in MM cell lines (MM.1S, OPM-2, NCI-H929, U266, and RPMI-8226) and normal plasma cells (nPCs). We concluded that the expression of MALAT1 was considerably increased in the 5 MM cell lines compared to nPCs cells (Figure 1B; P<0.05).

**Figure 1:** LncRNA MALAT1 expression in multiple myeloma (MM) **(A)** Relative expression of MALAT1 in plasma cells derived from bone marrow of healthy donors (Control n=19) and MM patients (n=37) were determined by qRT-PCR. **(B)** Relative expression of MALAT1 in normal plasma cells (nPCs) and MM cell lines (MM.1S, OPM-2, NCI-H929, U266, and RPMI-8226). ^**^ P<0.01; ^*^ P < 0.05.

### LncRNA MALAT1 inhibition suppressed MM cells proliferation

To further explore the role of MALAT1 in MM progression. MALAT1 shRNA was transfected into OPM-2 and U266 cell lines. QRT-PCR showed that MALAT1 expression was remarkably suppressed in sh-MALAT1 transfected MM cells (Figure 2A; P<0.05). CCK-8 assay showed that MALAT1 inhibition suppressed cellular viability of OPM-2 and U266 cells compared to sh-NC groups (Figure 2B; P<0.05). Colony formation assay also revealed that MALAT1 knockdown decreased MM cells clone numbers (Figure 2C; P<0.05). To determine whether the function of MALAT1 on cell proliferation was by altering cell cycle or apoptosis, flow cytometry assays were performed. Cell cycle analysis showed that MALAT1 knockdown induced MM cells cycle arrested in G0/G1 phase (Figure 2D; P<0.05). Apoptosis analysis indicated that MALAT1 inhibition enhanced MM cells apoptosis (Figure 2E; P<0.05).

**Figure 2:** Effects of MALAT1 on MM cells proliferation *in vitro* **(A)** Relative expression of MALAT1 in OPM-2 and U266 cells transfected with sh-MALAT1 or sh-NC. **(B, C)** The effects of MALAT1 on MM cells proliferation were determined by CCK-8 assay and Colony formation assay. **(D)** The effects of MALAT1 on MM cells cycle distributions were determined by Flow cytometry assay. **(E)** The effects of MALAT1 on MM cells apoptosis were determined by Flow cytometry assay. ^**^ P<0.01; ^*^ P < 0.05.

### LncRNA MALAT1 inhibition suppressed tumor growth *in vivo*

To further investigate the roles of MALAT1 on tumor growth *in vivo*. MM cells transfected with sh-MATAT1 or sh-NC were injected into the right scapula of mice. Xenograft tumors were examined 7 weeks after inoculation. Results showed that tumor volumes and weights in sh-MALAT1 group were significantly less than those in sh-NC group (Figure 3A-3C; P<0.05). Moreover, we used qRT-PCR to detect MALAT1 and miR-509-5p expression in tumor tissues. Results showed that MALAT1 expression was obviously decreased and miR-509-5p was increased in sh-MALAT1 group compared to sh-NC group (Figure 3D and 3E; P<0.05). In addition, immunohistochemical (IHC) staining showed that the number of Ki-67 positive cells in sh-MALAT1 group was obviously less than sh-NC group (Figure 3F; P<0.05). These data revealed that MALAT1 suppression could reduce tumorigenesis of MM *in vivo*.

**Figure 3:** MALAT1 knockdown inhibited tumor growth *in vivo* **(A)** The subcutaneous tumors were taken photos in sh-MALAT1 or sh-NC groups. **(B)** Tumor volume was measured every 1 week. **(C)** The subcutaneous tumors were weighted in sh-MALAT1 or sh-NC groups. **(D)** MALAT1 expression in tumor tissues was detected by qRT-PCR. **(E)** MiR-509-5p expression in tumor tissues was detected by qRT-PCR. **(F)** The expression of Ki-67 in xenograft samples was assessed by IHC staining. ^**^ P<0.01; ^*^ P < 0.05.

### MiR-509-5p expression was directly regulated by MALAT1

It has been elucidated that lncRNAs contain complementary sequences to miRNA. Based on this ground, they could be competitively binding to miRNAs and function as a competing endogenous RNAs (ceRNAs) [12]. Therefore, in the present study the bioinformatics tool DIANA was used to analyze MALAT1 targets, miR-509-5p was selected as the predicted target with the high score (Figure 4A). To confirm the direct target between MALAT1 and miR-509-5p, we constructed luciferase reporter assay. Our data showed that miR-509-5p mimics reduced luciferase activity of MALAT1-Wt, but not of MALAT1-Mut vectors (Figure 4B; P<0.05). To test this prediction, we determined the expression of miR-509-5p expression in MM samples. QRT-PCR showed that miR-509-5p expression was significantly downregulated in MM samples and negatively associated with the expression of MALAT1 in 37 MM samples (Figure 4C and 4D; P<0.05). Furthermore, qRT-PCR showed that MALAT1 inhibition significantly reduced the expression of miR-509-5p in MM cells (Figure 4E; P<0.05). However, overexpression of miR-509-5p did not affect MALAT1 expression in MM cells (Figure 4F; P>0.05).

**Figure 4:** MiR-509-5p expression was directly regulated by MALAT1 **(A)** The predicted binding sites between MALAT1 and miR-509-5p. **(B)** Dual-luciferase reporter assay revealed that miR-509-5p mimics decreased luciferase activity of MALAT1-Wt, but not of MALAT1-mut. **(C)** Relative expression of miR-509-5p in MM samples was determined by qRT-PCR. **(D)** Pearson's correlation analysis between miR-509-5p expression and MALAT1 expression in MM samples. **(E)** miR-509-5p expression in MALAT1 decreased MM cells was determined by qRT-PCR. **(F)** MALAT1 expression in miR-509-5p mimics transfected MM cells was determined by qRT-PCR. **(G, H)** RNA-IP assays were performed in MM cells transfected with miR-509-5p mimics and miR-NC. ^**^ P<0.01; ^*^ P < 0.05.

Previous studies showed that microRNAs degrade RNA or repress translation via an Ago2-dependent pathway [13]. Thus, in the present study, we used an anti-Ago2 RIP assay in MM cells transfected with miR-509-5p mimics. We found that endogenous MALAT1 was pulled down specifically in miR-509-5p overexpressed cells compared with sh-NC group (Figure 4G and 4H; P<0.05), indicating that miR-509-5p is a direct inhibitory target of MALAT1.

### MiR-509-5p reversed the effect of MALAT1 on MM progression

To further explore whether MALAT1 exerts biological functions through miR-509-5p, we used rescue experiments by inhibiting miR-509-5p expression in MALAT1 knockdown cells (Figure 5A; P<0.05). CCK-8 assay and clone formation assay showed that cell growth was reduced in MALAT1 suppressed MM cells, whereas miR-509-5p inhibitor partially reversed the reduction of cell proliferation ability (Figure 5B and 5C; P<0.05).

**Figure 5:** MiR-509-5p reversed the effect of MALAT1 on MM cell proliferation **(A)** miR-509-3p expression was determined by qRT-PCR in MM cells transfected with miR-509-5p inhibitor, sh-MALAT1. **(B)** Cell viability of MM cells were detected by CCK-8 assay. **(C)** Colony numbers of MM cells were determined by colony formation assay. ^**^ P<0.01; ^*^ P < 0.05.

### FOXP1 was the target of miR-509-5p and regulated by MALAT1

To identify the target of miR-509-5p in MM, TargetSCan was used to perform a target search, and FOXP1 came out as one of the best candidates (Figure 6A). Luciferase reporter assay showed that miR-509-5p mimics significantly reduced the luciferase activity of FOXP1-Wt, but not of FOXP1-Mut (Figure 6B; P<0.05). Western blot showed that miR-509-5p inhibitor increased FOXP1 protein expression in MM cells, while miR-509-5p mimics suppressed FOXP1 protein expression in MM cells (Figure 6C). Thus, these findings suggested that miR-509-5p might directly target the 3’-UTR of FOXP1 in MM cells.

**Figure 6:** MiR-509-5p directly targeted FOXP1 **(A)** Predicted binding sites for miR-509-5p in FOXP1 sequences. **(B)** Luciferase reporter assay revealed that miR-509-5p mimics decreased luciferase activity of FOXP1-Wt, but not of FOXP1-Mut. **(C)** FOXP1 expression was determined by western blot in MM cells transfected with miR-509-5p mimics and miR-509-5p inhibitor. ^*^P<0.05

To determine whether MALAT1 functions through FOXP1 mediated by miR-509-5p. We determined FOXP1 expression in MM samples by qRT-PCR. We found that FOXP1 expression was increased in MM samples compared to normal healthy controls (Figure 7A; P<0.05). Pearson's correlation analysis revealed that FOXP1 expression was positively associated with MALAT1 expression in 37 MM samples (Figure 7B; P<0.05). Furthermore, we determined FOXP1 expression (mRNA and protein) after MM cells transfected with sh-MALAT1 and miR-509-5p inhibitor. Our data showed that knockdown of MALAT1 significantly suppressed FOXP1 expression, whereas FOXP1 expression was rescued after introduction of miR-509-5p inhibitor (Figure 7C and 7D; P<0.05), indicating that MALAT1 regulated the expression of FOXP1 in a ceRNA manner and miR-509-5p played a key role in MALAT1-mediated regulatory.

**Figure 7:** MALAT1 regulated FOXP1 expression via miR-509-5p **(A)** Relative expression of FOXP1 in MM samples was determined by qRT-PCR. **(B)** Pearson's correlation analysis between FOXP1 expression and MALAT1 expression in MM samples. **(C, D)** Relative expression of FOXP1 mRNA and protein in MM cells co-transfected with sh-MALAT1 and miR-509-5p inhibitor. ^**^ P<0.01; ^*^ P < 0.05.

## DISCUSSION

MM is a neoplasm of terminally differentiated B cells (plasma cells), in which chromosome translocations frequently resulting in oncogenes formation under the control of immunoglobulin enhancers [2]. On a worldwide scale, it is estimated that about 86000 incident cases occur annually, accounting for about 0.8% of all new cancer cases [3]. Due to the rapid development of basic medical research, the molecular mechanisms underlying the tumorigenesis and pathogenesis of MM have been uncovered gradually over past few years. Increasing studies showed that dysregulation of lncRNAs might contribute to MM progression. For example, Sedlarikova et al found that lncRNA UCA1 was downregulated in multiple myeloma [14]. Meng et al found that lncRNA CRNDE promotes MM cell growth by suppressing miR-451 [15]. However, the function and underlying mechanism of lncRNAs in MM remain unclear.

The metastasis associated lung adenocarcinoma transcript 1 (MALAT1), also known as non-coding nuclear-enriched abundant transcript 2, has been identified to play important roles in alternative splicing, nuclear organization, and epigenetic modulating of gene expression [16]. A number of evidences indicate that MALAT1 was closely related to various pathological processes, especially cancer. For example. Zhang et al showed that upregulation of MALAT1 correlated with tumor progression and poor prognosis in clear cell renal cell carcinoma [17]. Wang et al found that MALAT1 promoted gallbladder cancer development by serving as a molecular sponge to regulate miR-206 [18]. Liu et al showed that down-regulation of MALAT1 inhibited proliferation and induced apoptosis in MM [19]. Furthermore, Cho et al showed that lncRNA MALAT1 was overexpressed in MM and might serve as a marker to predict disease progression [20]. However, the underlying mechanisms of MALAT1 in MM are still unclear. In the present study, our data showed that MALAT1 expression was substantially increased in MM samples and cell lines. *in vitro* assay, our data showed that MALAT1 suppression reduced MM cells proliferation, induced cell cycle arrest at G0/G1 phase and enhanced cell apoptosis. Furthermore, we showed that MALAT1 inhibition also suppressed tumor growth *in vivo*. These data indicated that MALAT1 might function as an oncogene in MM progression.

Recent studies have reported that lncRNAs exhibit the ability to act as a miRNA sponge and modulate the derepression of miRNA targets at post-transcriptional level [21]. For example, Wang et al showed that lncRNA XIST exerted oncogenic functions in human glioma by targeting miR-137 [22]. Zhang et al showed that lncRNA UCA1 promoted cell progression by acting as a competing endogenous RNA of ATF2 in prostate cancer [23]. Yang et al showed that lncRNA MIR31HG exhibited oncogenic property in pancreatic ductal adenocarcinoma and is negatively regulated by miR-193b [24]. In our study, we identified miR-509-5p as an inhibitory target of MALAT1 by sequence complementarity analysis and luciferase reporter assay. QRT-PCR showed that miR-509-5p was downregulated in MM samples and inversely corrected with the MALAT1 expression. QRT-PCR showed that miR-509-5p expression was decreased in MALAT1 knockdown MM cells. However, overexpression of miR-509-5p did not affect MALAT1 expression. In RNA-IP assay, we found that MALAT1 was significantly pulled down in miR-509-5p overexpressing cells. In addition, our data showed that miR-509-5p could reverse the effect of MALAT1 on MM growth. Therefore, these data indicated that miR-509-5p expression was directly regulated by MALAT1 in MM.

Forkhead box P1 (FOXP1) is a member of the forkhead box P subfamily, which consists of four members [25]. FOX family members are DNA-binding proteins which involved in transcriptional regulation and DNA repair and play critical roles in immune responses, organ development, and cancer pathogenesis [26, 27]. For example, Choi et al showed that FOXP1 functioned as an oncogene in promoting cancer stem cell-like characteristics in ovarian cancer cells [28]. Craig et al indicated that Myc-mediated repression of microRNA-34a promoted high-grade transformation of B-cell lymphoma by dysregulation of FOXP1 [29]. Halacli et al found that FOXP1 regulation via the PI3K/Akt/p70S6K signaling pathway in breast cancer cells [30]. Those studies suggested that FOXP1 play an important role in tumor progression. However, interaction between lncRNA and FOXP1 in MM is still unclear. In this study, our data showed that FOXP1 expression was increased in MM samples and positively associated with the MALAT1 expression. Furthermore, we revealed that MALTA1 could positively regulate the expression of FOXP1 by sponging miR-509-5p in MM cells.

In summary, our data showed that MALAT1 functioned as an oncogene, which played a major role in regulating malignancies in MM. In addition, we revealed that MALAT1 could modulate MM cell growth via targeting miR-509-5p/FOXP1 axis. Taken together, our data indicated that MALAT1 could serve as a potential therapeutic target for the treatment of MM patients.

## MATERIALS AND METHODS

### Primary MM samples

Thirty seven MM samples and nineteen healthy control samples were collected from April 2012 to January 2014 at the First People's Hospital of Shangqiu. Plasma cells were isolated from bone marrow samples as described previously [12]. The study was approved by the Ethics Committee of The First People's Hospital of Shangqiu and performed in accordance with the Declaration of Helsinki (2000). Written informed consent obtained from all patients.

### Cell lines and cell culture

We obtained MM cell lines (MM.1S, OPM-2, NCI-H929, U266, and RPMI-8226) and normal plasma cells (nPCs) from the American Type Culture Collection (ATCC, Manassas). Cells were cultured in RPMI-1640 medium (Invitrogen) supplemented with 10% fetal bovine serum (FBS, Invitrogen)and 1% penicillin/streptomycin at 37 C in a 5% CO_2_ atmosphere.

### Plasmid construction and transfection

miR-509-5p mimics, miR-509-5p inhibitor, lentiviruses short hairpin (shRNA) directed against MALAT1 (sh-MALAT1) and the empty lentiviral vector (sh-NC) were chemically synthesized from GenePharma Co., Ltd. (Shanghai, China). OPM-2 and U266 cells in logarithmic phase were transfected with miRNAs, sh-MALAT1, and their controls using Lipofectamine 2000 (Invitrogen) according to the manufacturer's instructions. Further experiments were carried out at 48 h post-transfection.

### Quantitative real time-PCR (qRT-PCR)

Total RNA in MM cells was extracted by using TRIzol reagent (Invitrogen) according to the manufacturer's instructions. High Capacity cDNA Reverse Transcription Kit (Applied Biosystems) was used to reversely transcribe RNA samples. And a miScript SYBR Green PCR Kit (Takara) was used for analyzing the expression of miR-509-5p, FOXP1 and MALAT1. Realtime-PCR was performed using the Applied Biosystems 7500 Sequence Detection system (Applied Biosystems). QRT-PCR reactions were performed using the following parameters: 95°C for 2 min followed by 40 cycles of 95°C, 15 s, and 60°C. All results were normalized to the expression of GAPDH or snRNA U6. 2^-ΔΔCt^ method was used for analysis of quantitative changes in gene expression according to the manufacturer's protocols. The primer sequences used are as follows: MALAT1 forward 5′-AAAGCAAGGTCTCCCCACAAG-3′, reverse 5′-GGTCTGTGCTAGATCAAAAGGC-3′; miR-509-5p forward 5′-TACTGCAGACAGTGGCAAUCA-3′, reverse 5′-GTGCAGGGTCCGAGGT-3’; FOXP1 forward 5’-TCCCGTGTCAGTGGCTATGAT-3’, reverse 5’-CTCTTTAGGCTGTTTTCCAGCAT-3’.

### Cell proliferation assay

The cell proliferation rate was detected using Cell Counting Kit-8 assays (CCK-8, Dojindo) according to the instructions. 100 ul cell suspension (1×10^3^ cells/well) was seeded in a 96-well plate and various concentrations of substances were added. The cells were incubated for an appropriate length of time (24, 48, and 72 h) and obtained with 10ul CCK-8 solution added. Absorbance was measured using a microtiter plate reader at 450 nm.

### Colony formation assay

Cells were plated in 6 well plates at a density of 600 cells/well and cultured for 8 days. The medium was changed every 3 days. Cells were fixed with methanol and stained with 0.2% crystal violet. After being washed mildly with PBS and air-dried, the visible colonies consisting of >50 cells were manually counted.

### Flow cytometry assays

For cell cycle analysis, at 48 h post-transfection, cells were harvested via trypsinization, washed with cold PBS and fixed in 70% ice cold ethanol overnight, followed by staining with 50 mg/ml propidium iodide (PI) for 30 min. For cell apoptosis analysis, cells were harvested and resuspended in fixation fluid at 48 h post-transfection. 5μl Annexin V-FITC and 2μl PI were added to 500 μl cell suspension. All cells were analyzed on the FACSCalibur flow cytometry (BD Biosciences). Data was analyzed using CELL Quest 3.0 software.

### Luciferase reporter assays

MALAT1 fragment containing putative or mutated miR-509-5p binding site was amplified by PCR and then cloned into a pmirGLO Dual-luciferase miRNA Target Expression Vector (Promega). The recombinant reporter vector was named as MALAT1-wild-type (MALAT1-Wt) or MALAT1-mutated-type (MALAT1-Mut). MALAT1-Wt or MALAT1-Mut was co-transfected with miR-NC or miR-509-5p mimics using Lipofectamine 2000 (Invitrogen). Luciferase assay was performed 48 h after transfection using a Dual-Luciferase Reporter Assay System (Promega).

Similar to above, the putative and mutated miR-509-5p target binding sequence in FOXP1 was synthesized and cloned into a luciferase reporter to generate the wild-type (FOXP1-Wt) or mutated-type (FOXP1-Mut) reporter plasmids. The transfection procedure was the same as described previously.

### RNA immunoprecipitation assay

RNA immunoprecipitation assay was performed using the EZ-Magna RIP RNA-binding protein immunoprecipitation kit (Millipore). All procedures were implemented following manufacturer's instructions. MM cells were lysed with RIP lysis buffer with RNase inhibitor, and subsequently incubated with RIP buffer. Antibody against argonaute2 (Ago2) (Millipore) was used to form conjugated magnetic beads. MALAT1 fold enrichment of RNA immunoprecipitation was normalized to the RIP fraction of control antibody IgG (Millipore), and was examined by qRT-PCR analysis.

### Western blot analysis

Cells were lysed with ice-cold lysis buffer. Proteins were separated with 10% SDS-PAGE and then transferred onto a PVDF membrane at 100 V for 1.5 h. Proteins were treated with TBS with Tween which contain 5% nonfat dried milk for 1 h. Blots were incubated with primary antibodies at 4°C overnight (FOXP1; ab16645, Abcam) followed by incubation with secondary antibodies at room temperature for 2h. After being washing with PBST, Blots were analyzed using Gel-Doc 200 (Bio-Rad). GAPDH was used as an internal reference.

### Tumor xenograft formation assay

Male athymic BALB/c mice, 5-week-old, were purchased from the Shanghai Experimental Animal Center of the Chinese Academy of Sciences. U266 cells were infected with sh-MALAT1 and sh-NC were subcutaneously injected into nude mice with dose of 10^7^ cells per mouse. We monitored the primary tumor growth by measuring tumor sizes each week after injection. Tumor volume was estimated with the formula, volume= 0.4 X length X Width^2^. All animals were sacrificed 7 weeks after injection. The tumor tissues were excised, treated with formalin and embedded with paraffin for further analysis. All procedures were performed in accordance with the National Institutes of Health Guide for the Care and Use of Laboratory Animals.

### Immunohistochemistry

Immunohistochemistry (IHC) was performed on formalinfixed, paraffin-embedded mouse subcutaneous tumors. Tissue sections were deparaffinized, rehydrated, and heat- induced antigen retrieval was performed in an autoclave in 10 mM citrate buffer (pH 6.0) for 5min. Endogenous peroxidase activity was blocked with 0.3% hydrogen peroxide for 15 min. Sections were incubated with anti-Ki-67 at 4 °C overnight. Tissue sections were then incubated with secondary antibody for 30 min.

### Statistical analyses

Statistical analysis was carried out by the SPSS 18.0. Data was described as mean±standard deviation (SD). The quantitative data between groups was compared and analyzed by Student's t-test or one-way ANOVA. P<0.05 was considered as statistically significant. Each experiment was repeated at least three times.
